# Phenotypic Screening of Molecular Docking Enriched Chemical Libraries from Targets Identified in Ischemic Stroke Genome Data by Network-Based Method

**DOI:** 10.1155/2021/9999340

**Published:** 2021-11-15

**Authors:** Xiaojiang Peng, Dao-jin Xue

**Affiliations:** ^1^Zhaoqing Medical College, No. 6 Xijiangnan Road, Duanzhou District, Zhaoqing 526020, Guangdong, China; ^2^The Second Affiliated Hospital of Guangzhou University of Chinese Medicine, Guangdong Provincial Hospital of Chinese Medicine, 111 Dade Road, Yuexiu District 510120, Guangzhou, China

## Abstract

Cerebral ischemia (IS) is one of the main cardiovascular diseases threatening life and disability. Like most cardiovascular events, the disease progression of is affects a variety of signaling pathways and changes multiple overexpressed genes in the body. The use of new therapeutic agents to interfere with the disease progression of cardiovascular diseases (such as is) can be achieved by selectively regulating small molecules of the target set of different signal pathways, also known as selective multipharmacology. Phenotypic screening can be an effective method to solve this problem, but the lack of targeted methods for ischemic stroke limits its impact. Here, we aim to identify IS-specific targets by RNA sequencing data with a network-based approach. Molecular docking approach was applied to screen over 210,000 molecules from SPECS compound library. Screening of this enriched library resulted in 605 candidates that led to several potent active hits. The novelty analysis suggested that the structure scaffolds of the compounds were dissimilar to existing IKKB inhibitors, and further biological test result confirmed two identified compounds represented novel IKKB inhibitors. Further, docking exploration with IKKB (PDB id: 4KIK) showed that the three selective compounds were stable inside the binding pocket of IKKB which shared a homology of compound-protein interactions in comparison with the bioactive inhibitor of CHEMBL1762621. Our screening method is expected to produce selective multidrug lead compounds for the development of treatments for complex diseases, such as ischemic stroke.

## 1. Introduction

Cerebral ischemia (IS) is the most destructive manifestation of atherosclerosis and systemic hypertension. It is the second highest source of death and the third leading source of disability across the world [1]. At slightly over 16 million 900 thousand cases, the disease has a relatively high incidence rate globally [2]. Based on previous studies, the primary causes of the stroke are inflammation, atherosclerosis, blood coagulation, and platelet activation [3]. The use of rapid chemical and rapid mechanical thrombolysis following stroke incidence is considered a traditional treatment method. These interventions require immediate treatment and therapy Also, the risks of intracranial hemorrhage and other forms of bleeding have been observed in heightened thrombolysis [4]. Consequently, the immediate detection of ischemic stroke events by serum biomarkers may have important clinical value for disease prevention, treatment, and prognosis. Currently, the treatment and detection of IS is largely based on cardiac tomography imaging, including a reliance on computed tomography as well as magnetic resonance imaging (MRI) [5]. Ultimately, identification of potential therapeutic agents for the prevention, detection, and treatment of cerebral ischemia is overly important.

While the diagnosis of myocardial infarction is usually based on the use of ECG, contemporary studies appreciate the significance of circulating RNAs in the detection of the dysregulated genes in chronic ischemic stroke. In particular, the stability of blood samples coupled with perceived feasibility of detection renders them to be valuable genomic data [6]. In the past, studies applied differential expression analysis in the identification of the miRNAs that were differentially manifested following probe sequencing. However, this method is limited in its focus on the responsibility of a single target and thus fails to deal with the complex disease like ischemic stroke; thus, we seek to build the relationship between genes in a network perspective and establish the relationship between genes and diseases for the purpose of polypharmacology. This problem can be solved by a network-based approach of target identification from enormous genomic data with weighted gene coexpression network analysis (WGCNA) [7].

Nowadays, applying genomic and structural protein data into the discovery of novel therapeutic agents was in trend as it enhances the efficiency and accuracy of target identification. L1000 was a comprehensive genetic map based on the perturbation of compounds to disease and genes [8]. Here, we follow a combination approach with network-based approach of target and phenotypic screening to generate novel molecules with selective polypharmacology that may have potency in treating ischemic stroke.

Our approach combines disease-related targets selected by genomic profiles as well as binding site identifications to come up with several targets with druggable binding pockets [9]. An estimate of 210,000 compounds from SPECS library is docked against every disease-related targets [10]. Minute molecules whose prediction is to simultaneously bind on several proteins are identified and selected for phenotypic screening using molecular docking. The impact of the compound on IKKB is also tested based on an inhibition activity assay [11]. In uncovering probable approaches of action, the compounds were identified for docking to the IKKB protein complex in comparison with the bioactive agents.

## 2. Materials and Methods

### 2.1. Genomic Data Preparation of Ischemic Stroke

The current study uses IS gene expression data sourced from the GEO's genomic database. Gene annotation was extracted with the resultant data being retrieved such as Entrez ID as well as gene symbols and based on an inherent reference to the platform GPL570 (Illumina Inc.). In an effort to ensure the comparability and integrity of the selected data sets, a calculation of normalization with log 2 manifestation is made with RMA package. The mapping of the gene annotation in the identical gene symbol corresponding to multiple probes is made with the probe with the biggest mean manifestation across all samples. Consequently, the expression matrix of the samples is mixed up based on the miRNA/gene symbols. All the samples are then tested in an effort to alleviate the batch effect through reliance on the SVA toolkit.

### 2.2. Differential Expressed Gene Screening

Following the elimination of the abnormalities and duplicate, the normalization of differential expressed genes was done and calculations with package DEseq made. Lastly, genes with *p* value below 0.05 and foldchange >1 were identified for more network analysis.

### 2.3. Establishment of WGCNA Network and Detection of Disease-Associated Genes

The processing of data is achieved using WGCNA tool in RStudio 3.6.0 software. In safeguarding reliability in network construction, the researchers eliminated abnormal genes. Initially, a selection of the soft threshold of network construction is made to ensure the continuity of the adjacency matrix from 0 to 1, such that the constructed network is consistent with the power-law distribution. This process also ensures that it maintains closeness with the actual state of biological network. The construction of the scale-free network is dependent on the block module function, before carrying out the module partition analysis and determining coexpression module of the gene; then, the clustering and pairing of genes that have similar expression patterns is done. Through a reliance on the dynamic algorithm, the clustered tree is divided into branches to facilitate modules definitions, and modules then are assigned across different colors for better visualization. All the modules are summarized using module eigengene (ME). The modules are identified through their most significant module eigengene (ME) and are determined as a symbolic gene that represents the manifestation spectrum of all genes within a specific module. The definition of module membership (MM) is based on the correlation between module eigengene and individual gene. Moreover, the calculation of gene significance (GS) within the module is conducted to represent the correlation among traits and genes.

### 2.4. Protein Structures Acquisition

Gene ensemble IDs from the module with highest disease-correlation were converted to gene symbols via the ID converter tool from David website. Converted gene symbols were mapped to protein identifiers using the web interface of mapping tool provided by UniProt (http://www.uniprot.org/mapping). An annotated set of 594 reference human proteins were acquired from UniProtKB/SwissProt. FASTA sequence of each protein was retrieved for further alignment with the structures in the RCSB Protein Data Bank (PDB). The FASTA sequences were first queried against the pdbaa dataset using BLASTTP (protein-protein BLAST v2.10.1). To minimize the searching scope to find the protein structures with significant sequence identity to the query, only structures with *E*-value <10-5 and >90% sequence identities were kept. The identified structures were scrutinized for the experiment methodology, taxonomy for each structure chain, and the structure resolution to determine that the structures were from X-ray diffraction. The filtered criteria for crystal structures were with a resolution less than 3 angstrom (Å). To reduce redundant structures identified from BLASTTP and generate a set of representative structures related to each queried proteins, the CD-HIT (v4.8.1) was introduced for clustering the protein sequences of identified structures, and the threshold of similarity was set as 0.7 with identity over 90%, after which the cluster centers from CD-HIT were used as representative sequence for binding sites identification on the basis of structures. In total, 22 proteins that had one minimum crystal structure were identified.

### 2.5. Binding Site Identification

For each cluster identified by CD-HIT, the cluster centroid protein structure was further used for binding sites identification. The sitemap module in Schrodinger software suite was incorporated to identify the druggable binding sites on the crystal structures. The single chain of protein structures was acquired from PDB, and the binding ligands were removed to acquire the monomeric representative structures. Solvent molecules and bound ligands and any other heteroatoms were removed, and selenomethionine residues were substituted with methionine. The Protein Preparation Wizard workflow was further introduced for the preprocessing of monomeric structures. Missing loops and side chains were summed using Prime module. Disulfide bonds were then added, and each crystal structure was protonated with PROPKA at pH 7.0. Binding sites were identified in SiteMap with the processed protein structure. For each structure, 10 binding sites were kept, with all the other parameters unadjusted. The binding sites with Site score and Drug score over 0.9 were kept. The average coordinates of the sitemap spheres were defined as the centroid of the binding site. Binding sites with a Drug score above 1.0 were identified as druggable. In total, 192 druggable binding sites were identified for 22 proteins.

### 2.6. Inferring the Binding Sites

All binding sites were evaluated in response to the contact surface, H-bond donor/accepter, enclosure, hydrophilic/hydrophobic score, and the binding site size and volumes for the identified proteins, to keep only the most druggable binding sites. The result showed that 19 druggable binding sites from 12 proteins were evaluated as the most druggable. To determine the biological activities of all binding sites, functional annotation for all proteins was performed and grouped accordingly. The ratio of proteins belonging to identical functional group was calculated. All binding sites were with bioactive ligand in reference to complex structure from PDB.

### 2.7. Molecular Docking

All molecular docking studies were performed with the Schrodinger Software. The docking method was as described. 210,070 compounds from SPECS database (obtained in July 2019) were prepared for ligand-protein docking. The crystal structure (PDB ID: 2ZVN, 3BRT, and 3BRV) was used to build the energy grid, which was generated at the centroid of the most druggable binding sites. The protocol constraints including QikProp and Lipinski filter were employed to determine compounds with suitable pharmacological properties. Glide HTVS scoring function was tested to evaluate the binding affinity of compounds, and further compounds were ranked by predicted scores. Compounds ranked at the top 0.1%, 0.1%, and 0.05% with good scoring were filtered with XP, accordingly. All other parameters were set as default settings in the grid generation and docking.

### 2.8. Novelty Test of Compounds

Compounds ranked at the top 0.1% and 0.05% from docking were compared with biologically active compounds from bioactive inhibitor of CHEMBL1762621 from CHEMBL24. Generally, the compound structures were converted to Canonical Smile string, and transformed to Morgan fingerprints with the OpenBabel node from Knime. The novelty of compound was defined with a Tanimoto similarity (Tc) score lower than 0.2.

## 3. Results

### 3.1. WGCNA Network Construction and Identification of Disease-Related Modules

One of the obvious advantages is that WGCNA clustered genes into coexpression module, which served as a network-based target identifying method on RNA-seq data, and it has been proved as an effective application in bionetworks, capturing gene, and disease-related traits with high sensitivity to low abundance without losing much information [12]. Previous studies have shown that WGCNA provides important modules and pathways for many diseases [13–15] and solved the problem in identifying coding genes that play a key role in cancerous and neurodegenerative diseases as well [16, 17]. The preliminary purpose of this step is to identify ischemic stroke-specific genes based on the adjacency network between gene modules established by the method of WGCNA [18]. This finding may help in identification of disease-related modules.

Gene expression profiles (GSE26887) were collected for IS patients from public open-source database of GEO. A total of 20 IS and 20 normal samples have been annotated with references to the sequencing platforms of Affymetrix. The genomic data were used to perform weighted gene correlation network analysis to identify disease-related gene modules that are correlated with the disease features in ischemic stroke (*p* < 0.001, FDR < 0.01, and |log2fold change| (log2FC) > 1) (Figure 1). In total, 141 genes were identified as disease-related genes in IS patient samples.

In this study, a total of 4838 genes were screened to establish the network. After removing the deleted and abnormalities, the genes were screened for subsequent analysis. The network construction parameters were defined when the soft threshold power is adjusted to 6 to reach the scale-free topological index of 0.9 (Figure 1(a)). Linear recession of scale-free topology to log10 of *k* showed a robust correlation (Figure 1(b), *R*^2^ = 0.87). Therefore, the network is closer to the real biological network state as the node degrees in the biological network follow a power-law distribution [19].

The heatmap shows the disease-gene adjacency matrix of the modules. The resulting gene tree and corresponding module colors are shown in Figure 1. There were 12 ischemic stroke (IS) disease features (age scale, sex, percentage of hypertension, percentage of smoking history, percentage of hypercholesterolemia, percentage of obesity, percentage of diabetes mellitus, family history, total cholesterol, high-density lipoprotein (HDL) level, and infraction volume), and the Framingham score [20] was correlated with the gene expression level with WGCNA to identify the IS-specific genes (Figure 1). Our network was based on the genomic data of over 4000 genes from 40 samples; the result showed the turquoise module exhibited a correlation coefficient of 0.88 with the Framingham score calculated. Thus, the turquoise module was identified as the IS disease-related module (*p* value =1.8*e* − 12). Using our approach, the genes in the disease-related module were identified for selection of ischemic stroke-related targets.

### 3.2. Identification of Ischemic Stroke-Specific Gene and Disease-Related Targets

The use of target identification in present implementations among phenotypic screening in complex disease is highly limiting. The current study proposes a strategy that utilizes genomic profiles from ischemic stroke in phenotypic screening. This process starts through the detection of druggable pockets within sets of disease-specific protein structures sourced from the Protein Data Bank (PDB). We searched for translation products encoded by the 141 disease-specific genes and clustered the protein sequences with CD-HIT to eliminate similar sequences with threshold of 90%, so as to find the representative disease-specific proteins by assigning cluster centroid [21]. Druggable binding sites were predicted based on the SiteMap program on the disease-specific protein surface and further evaluated its druggability via Drug Scoring and Site Scoring [22].

We look into the result of the disease-related module of IS; 141 disease-related genes with elevated gene significance (GS) and module membership (MM) were further identified for subsequent disease-related targets identification. An analysis from the 20,192 reference proteins based on UniProt/kB [23] identifiers resulted in 594 proteins that were encoded by the disease-related genes. For every gene, the study identified with protein products has at least one high-resolution crystal structure by mining the Protein Data Bank (PDB). A total of 594 unique protein chains with a minimum of one crystal structures from the PDB mapped to the 141 disease-related genes.

The set of 594 protein sequences that encoded the disease-specific genes were obtained from the UniProt database. Subsequently the sequences were aligned to decide the sequence similarity with the others. The encoding proteins the disease-related genes implicated in IS disease-specific module were clustered with CD-HIT to acquire the cluster centroid as representative structure with a threshold of 0.9. Among the 594 previously identified disease-specific proteins implicated in ischemic stroke, a total of 22 cluster centroids were identified in the proteins. In total, 22 clusters of the 596 proteins were identified and 22 proteins were regarded as the disease-related proteins.

### 3.3. Annotation of Binding Sites of the Disease-Related Targets

The study used the three-dimensional structure of disease-related protein for ischemic stroke to scan the surfaces for potential binding sites through the SiteMap program. This program selects binding sites through imposition of a 3D grid across the entirety of the protein, thus determining the energies of van der Waals on every point in the grid (site point). Through linkage of site points across the protein surface protected against the solvent, the program detects probable binding sites within protein surfaces. All binding sites detected in the program are evaluated for their druggability (Drug score) and their ability to bind a ligand (Site score). The ability to bind a ligand reduces the effect of hydrophilicity in highly polar and charged sites. Binding sites that have with DrugScore and SiteScore of 0.8 are perceived to be able to fit small molecule ligands. In contrast DrugScore and SiteScore values that are closer to 0.8 are perceived “difficult” to drug. On the other hand, binding sites with DrugScore and SiteScore values that are closer to 1.1 are considered to be overly “druggable.” In the current study, binding sites with DrugScore and SiteScore values of 0.9 or greater are selected for probing and binding sites with DrugScore above 1.0 are considered to be druggable. In summary, 19 pockets in 12 proteins were identified as druggable binding pockets of the disease-related proteins.

To further validate the protein family of the disease-related proteins, p-fam database with a hidden Markov model was used to decide the protein families [24]. The result indicated the 22 disease-related proteins were assigned into 3 major families including NEMO, gelsolin, and serpin (Figure 2). The top-ranked protein family of NEMO with the highest ratio of disease-related proteins was applied for further compound-docking identification with the cocrystallized structure of the disease-related proteins (PDB ID 2ZVN, 3BRT, and 3BRV).

### 3.4. Docking of Compounds from SPECS Chemical Compound Library

To identify small molecules that inhibit disease-specific proteins with IS, a chemical compound library of SPECS with approximately 210,000 compounds was docked to the druggable binding sites identified on structures of disease-specific protein (PDB id: 2ZVN, 3BRT, and 3BRV). The number of druggable binding sites with Drug Scoring and Site Scoring better than a given cutoff of 1.0 and 0.9 of all compounds in the library was used. In this work, scoring cutoff corresponding to a computational binding free energy lower than −6.5 kcal/mol was used. For compounds docked to 2ZVN, 3BRT, and 3BRV. Approximately 30% of the compounds were predicted to bind to the binding sites of 2ZVN, 14% of the docked compounds were predicted to bind to 3BRT and 8%, and 3BRV in the HTVS mode of docking (Figure 2). Less than 0.1% (238), 0.1% (230), and 0.05% (137) of the compounds were predicted to bind to 2ZVN, 3BRT, and 3BRV with a good scoring of binding free energy (Figure 2), respectively.

Small molecules with a good scoring of predicted binding free energy of ischemic stroke-related targets (2ZVN, 3BRT, and 3BRV) were identified for more testing. About 605 compounds were identified based on their prediction to target across the three IKKB proteins on the identified binding sites. The average value across predicted compounds for each target is about 200. The top scoring compounds were grouped based on hierarchy through reference to chemical similarity. For every cluster, the corresponding compounds were qualified for phenotypic testing. Docking with Schrodinger software suite scoring model was utilized in predicting the binding affinities for every pair to evaluate the interactions between protein and compound.

### 3.5. Novelty Analysis of Compounds to Targets

To further investigate the novelty of the compounds, the pairwise similarity between the tested compounds and bioactive IKKB inhibitors in the CHEMBL24 was calculated based on the Morgan fingerprints using the fingerprint similarity node from Knime. The Tanimoto coefficients (Tc), ranging from 0 (complete dissimilarity) to 1 (identical), were employed to compare the chemical similarity between each molecule pairs [25]. A pair of molecules with chemical dissimilarity have low Tc value close to 0, whereas identical pairs possess a Tc value equal to 1. About 95.2%, 98.3%, and 100% of the docked compounds, found to be potent inhibitor of IKKB, were all less than 0.2. Hence, the novel chemotypes identified from virtual screening were reflected by their low Tc values and are expected to be promising novel candidates for IKKB.

### 3.6. Biological Activities

The three screened compounds based on the molecular docking with 4KIK evaluated the inhibition activities against IKKB with purchased Elisa kit. CHEMBL1762621, a bioactive IKKB inhibitor was used as control. The preliminary in vitro assay indicated that of the three selected inhibitors, 7378 displayed promising inhibition potency against IKKB. Compound SPECS230-7890 also displayed comparable inhibition activity against IKKB in the comparison with the known IKKB inhibitor CHEMBL1762621. Moreover, compound 7378 showed stronger inhibition against IKKB than CHEMBL1762621. This implies that our phenotypical screening approach may be considerable in filtering novel compound with bioactivity.

### 3.7. Exploration of Molecular Binding Mode of Compounds

To explore the interactions of compounds on IKKB, molecular docking with SP mode in the Schrodinger program were performed. The study then examined the binding modes of compound for every target as predicted by the docking scoring function. Every target was then classified based on the binding site's structural context through results of SiteMap as well as the protein's functional context. The binding modes of 7378 were at binding sites inside the enzymes' active sites. Three binding sites were next to predicted binding pockets of the ligand of IKKB.

Further, we prepared IKK-beta protein complex proteins for the docking calculation. CHEMBL1762621 is an active inhibitor for IKKB, and its IC50 for IKKB is submicromolar. We chose CHEMBL1762621 as control molecules to explore the mechanism responsible for the interactions between the selected compounds and IKKB. We performed docking of inhibitor CHEMBL1762621 to the X-ray crystallographic structures of the stable IKKB protein (PDB ID 4KIK). Similarly, 7378 and other 2 compounds were predicted to bind to sites adjacent to the active sites on 4KIK. The compound was predicted to bind with a similar pattern at the protein-ligand interfaces at binding pocket of 4KIK. In our docking studies, 7378 had a similar docking position against IKKB, providing the same result as CHEMBL1762621 against the same receptor. The predicted binding energy in the docking studies for 7378 was stronger than CHEMBL1762621 against IKKB (−7.182 kcal/mol). The binding energy of compound 7890 and 27964 was −7.06 and −6.21 kcal/mol against IKKB, which implied that both compounds possessed a stronger affinity for IKKB than CHEMBL1762621 (−3.183 kcal/mol). Compared with the bioactive inhibitor CHEMBL1762621, the compounds 7378, SPECS230-7890, and SPECS230-27964 were stabilized inside the binding pocket of IKK-beta protein, resulting in good affinity against IKK-beta. In the compound CHEMBL1762621-IKKB complex, the hydrogen bonded to the side chain … of Glu612 and Ser611, *π* − *π* stacking interaction with … Additionally, the ligand was predicted to form van der Waals interaction with residue. These interactions were maintained from the docking to IKKB with 7378.

## 4. Discussion

Coronary artery diseases, such as ischemic stroke, exhibit multiple phenotypes that include inflammation, atherosclerosis, blood coagulation, and platelet activation [2]. The phenotypes were largely impacted from gene perturbations as well as their transcription products that work in association with several signaling pathways. All the numerous targets promoting inflammation, atherosclerosis, blood coagulation, and platelet activation in ischemic stroke (IS) progression pose an impending problem to the progression of small molecule therapeutic agents that cure the disease. Today, the most popular strategy of drug discovery for coronary artery disease is to establish minute molecules to modulate functions in single targets. The concept has contributed to little novel therapeutic compounds that are effective against complex cardiovascular disease like IS. Nowadays, phenotypic screening is used in the discovery of drug to find novel therapeutic compounds. Phenotypic screening thus results in approval of several drugs, but the limitation in diversity of chemical libraries as well as the reliance on in vitro cell lines, coupled with curation of large bioassays datasets has always led to poor activity, thus yielding little efficacy among patients.

A data-based strategy combining protein-ligand, structural, and genomic interaction data in enriching chemical libraries with molecular docking reveals the prospect of hurdling the limits for phenotypic screening in facilitating drug discovery within coronary artery disease. The study applied a screening strategy integrating voluminous orthogonal datasets, such as (i) ischemic stroke genomic data derived from patient records at GEO, (ii) 3D structures of proteins enabling the detection of druggable pockets with sitemap in proteins implicated in ischemic stroke, and (iii) the predicted protein-ligand interactions using docking method. Particularly, the current approach first utilized data expression from GEO to identify disease-related gene modules with good scoring of gene significance and module membership. The PDB is successively mined to select existing protein structures, which are encoded by the genes. The study used CD-HIT in clustering these proteins by its sequences. Druggable pockets across the structures are detected for use in structure-based screening that identifies probable small molecule inhibitors. The proteins that have enrichments in the protein family (p-fam) for involvement in protein-ligand engagements and contain druggable pockets have uses in structure-based docking of a chemical entity library of SPECS with over 210,000 compounds. The affinity scoring of protein-compound complex were grouped to select the top ranked 0.1% molecules that bind to the IS-specific proteins. The resultant compounds are tested for pairwise similarity with the bioactive drugs from CHEMBL utilizing Tanimoto coefficient (Tc) scoring function by comparing chemical descriptions like Morgan fingerprints, and bioassays and molecular docking were performed to explore the binding poses and protein-compound interaction. The current strategy poses inherent benefits compared to conventional phenotypic screening because libraries with enormous compounds have the potential for rapid enrichment to identify small collections for candidates. The molecular docking was further performed to explore the mode of action of compounds.

Molecular docking was further utilized in uncovering a prospective approach for compound 7378. Protein function annotation uncovered potential targets of 7378, including IKKB. A specific target (IKKB) was one of the targets of 7378 that came out of the structure-based docking analysis. An evaluation of the predicted binding mode shows that these compounds can bind on the catalytic site in the structure. It may be true that targets other than IKKB show direct binding with 7378. Furthermore, IKKB is a key regulating protein for signaling transduction that interacted in various protein to protein engagements. Even though the study confirmed the binding to IKKB, it failed to establish whether the compound directly limits IKKB upstream or downstream signaling transductions. Still, the designing of the compound was based on the selective binding across many targets, and it is likely that target redirection or binding on other targets will happen. Furthermore, technical experiments beyond the context of the current study are necessary in exploring the specific workings of the compound.

In the recent past, multiple signaling pathways associated with regulation of tumor have been confirmed to relate to heart disease, including mTOR-Akt signaling pathway [26], JAK-STAT signaling pathway [27], and NF-*κ* B (NF-*κ* b) signaling pathway [28], which has a significant role in the progression of tumors associated inflammatory response. There is an association between the hyperactivation of NF-kB within cells and cancer, inflammation, and other human diseases [29].

The nuclear factor *κ*B (NF-*κ*B) is localized within the cytosol after complexion with I*κ*B*α*. The core elements of NF-kB cascade may control the translocation and activation of NF-kB transcription factor. Proinflammatory stimuli phosphorylate the IKK*β* subunit of I*κ*B*α* kinase (IKK) complex, thus causing its activation [30]. Activation of IKK now phosphorylates I*κ*B*α* results in its degradation and consequent release of NF-*κ*B, which is translocated to the nucleus to work as a factor of transcription. IKK*β* has a significant role in ischemia-induced brain damage [12, 31–38]. It further functions as a regulator of vascular stability and is a therapeutic target for cancer and inflammatory ailments. Thus, significant effort has been committed to identification of minute molecules inhibiting IKK*β* in the treatment of ischemic stroke. Our screening method is expected to produce selective multidrug lead compounds for the development of treatments for complex diseases, such as ischemic stroke.

## Figures and Tables

**Figure 1:** Construction of the weighted-gene correlation network. (a) Histogram and dot plot of the scale free topology scale of *k* of the disease-related gene network. (b) Dendrogram plot of clustered disease-related modules with hierarchy tree view and colors. (c) Heatmap of characteristic gene adjacency. The color bars on the left and below indicate the modules for each row or column.

**Figure 2:** Filtering compounds from SPECS library to targets implicated in ischemic stroke by docking to pockets identified by SiteMap of IS-specific druggable proteins. (b) Histogram showing number of compounds docked to predicted IS-specific targets. (c–e) Histogram plots portraying the rate of compounds that are predicted to bind the IS-specific targets of 2ZVN, 3BRT, and 3BRV, respectively. (f) Pangram of filtered 605 compounds to IS-specific targets.

## Data Availability

The original data for this study will be provided upon request after publication.
